# Harnessing Therapeutic Potentials of Statins Using Nanofibrous Carriers

**DOI:** 10.1155/2021/7265505

**Published:** 2021-11-02

**Authors:** Mahshid Ataei, Basil D. Roufogalis, Prashant Kesharwani, Tannaz Jamialahmadi, Amirhossein Sahebkar

**Affiliations:** ^1^School of Pharmacy, Mashhad University of Medical Sciences, Mashhad, Iran; ^2^Department of Toxicology and Pharmacology, School of Pharmacy, and Toxicology and Diseases Group, Pharmaceutical Sciences Research Center, The Institute of Pharmaceutical Sciences (TIPS), Tehran University of Medical Sciences, Tehran, Iran; ^3^Discipline of Pharmacology, School of Medical Sciences, University of Sydney, Sydney, NSW, Australia; ^4^National Institute of Complementary Medicine, Western Sydney University, Westmead, NSW, Australia; ^5^Department of Pharmaceutics, School of Pharmaceutical Education and Research, Jamia Hamdard, New Delhi 110062, India; ^6^Department of Nutrition, Faculty of Medicine, Mashhad University of Medical Sciences, Mashhad, Iran; ^7^Biotechnology Research Center, Pharmaceutical Technology Institute, Mashhad University of Medical Sciences, Mashhad, Iran; ^8^Applied Biomedical Research Center, Mashhad University of Medical Sciences, Mashhad, Iran

## Abstract

Statins are a wide category of 3-hydroxy-3-methylglutaryl-coenzyme A (HMG-CoA) reductase inhibitor drugs extensively prescribed for hypercholesterolemia. In fact, many studies showed beneficial effects of these agents on a variety of related illnesses, which include increased atherosclerotic plaque stability, decreased proliferation of vascular smooth muscle, platelet aggregation, the dampening of vascular inflammation, and also anabolic effects on bone tissue. Therefore, these drugs are considered as pleiotropic agents having different clinical applications other than those for which they were initially developed. Controlled drug delivery is an efficient way of delivery in tissue engineering. Amongst different controlled release formulations, nanofibers are a novel, alternative, widely used agent because of their unique properties. These include their sustained release of drug, a high drug-loading capacity, flexible shapes with a high surface-to-volume ratio, and superior porosity. Electrospinning is an economic and a simple method employed to produce nanofibers. In this report, studies related to statin nanofiber applications have been reviewed and their results have been summarized. Four different applications of statin nanofibers have been reported, including bone generation, endothelial stenosis and thrombosis, peripheral nerve injury, and anti-inflammatory action. Studies carried out both in vitro and in vivo showed effectiveness of statins in bone healing, aneurysm, and the healing of sciatic nerve injury. In addition, statins showed apoptosis effects and anti-inflammatory effects, with dose-dependent reduction of IL-6 and dose-independent reduction of TNF-*α*. Despite these promising results, validation via clinical trials is yet to be performed. The scope of statins in their pleiotropic range of actions is still not completely explored, and studies are still needed to enlighten different useful aspects of such drugs.

## 1. Introduction

The 3-hydroxy-3-methylglutaryl-coenzyme A (HMG-CoA) reductase inhibitors (statins) have been in use for more than 30 years to decrease the rate of occurrence of coronary artery disease and stroke. Despite the introduction of newer agents [1–3], statins are mostly prescribed for hypercholesterolemia because of their effect in reducing LDL [4]. Statins inhibit isoprenoid important lipid attachments, which are crucial for intracellular signaling of molecules like Rho, Rac, and CDC42 [5]. In cell culture and from animal studies, these effects have been shown to alter the expression of endothelial nitric oxide synthase, increase the stability of atherosclerotic plaques, and enhance the reactivity of platelets and production of proinflammatory cytokines and reactive oxygen species, along with effects on development of cardiac hypertrophy and fibrosis [6]. The results obtained from these studies demonstrate that statins in general have cholesterol-independent activities [5, 6]. In fact, statins are pleiotropic agents with different clinical applications [7–13], the action of which can be related or unrelated to the basic mechanism involved. These effects may be beneficial (such as the inhibition of HMG-CoA reductase) or neutral or even cause unwanted effects like toxicity and other related side effects [14, 15]. Major beneficial effects of statins include improvements of endothelial function and blood flow with increased stability of atherosclerotic plaques and inhibition of vascular smooth muscle proliferation and platelet aggregation, with overall dampening of vascular inflammation [16]. In addition, statins have been shown to improve arrhythmias (atrial fibrillation and ventricular tachyarrhythmias) [17]. Additional actions are induction of an anabolic effect on the bone tissue [18]. Several preclinical studies suggested that statins can inhibit tumor growth and also induce apoptosis in specific types of cancer [19].

There are several methodologies which can be employed to alleviate the effects of neointimal hyperplasia. Amongst them, the new drug-eluting stents (DESs) have a significant potential in reducing this condition. Therefore, use of stents and statins for coronary artery disease (CAD) is common with statin treatment, consistent with their lipid-lowering, antioxidative actions, and anti-inflammatory and antithrombotic effects useful for treating patients at different stages of the CAD disease [20].

Another effect of statins is their potential for osseointegration. Studies have shown the effects of statins on the activation of osteoblasts and reduction of osteoclasts both in vivo and in vitro, along with increased expression of bone morphogenetic protein-2 (BMP-2) [21], following inhibition of the mevalonate pathway [22]. Furthermore, recent studies have revealed that statins generally increase the expression of vascular endothelial growth factor (VEGF) [21]. In addition, the concentration of osteoprotegerin- (OPG-) binding protein, a soluble homodimer which is secreted from the osteoblasts, is highly increased after bone injury. It also antagonizes the receptor activator of nuclear factor-*κ*B ligand (RANKL), a known osteoclast formation molecule. Statins simulate the production of OPG and as a result, they are recommended as bone generator and integrator agents [21, 22].

Electrospinning is simple, economical, and versatile and provides a method in which polymer solution or melt undergo stretching and elongation through electrostatically driven jets, thereby forming polymer nanofibers (NFs). This method consists of three main parts including a source of high voltage, a syringe pump, and a conductive collector [23]. The diameter of these NFs ranges from nanometers to micrometers, and they are generally prepared using pharmaceutical and biodegradable polymer [24, 25]. These NFs characteristics are controlled by various parameters, including the solution characteristics, controlled variables, polymer properties, and processing variables such as applied voltage, distance, temperature, and flow rate [26]. Most recently, this method is mostly used for loading drugs for use as a novel drug delivery system (DDS).

Controlled drug delivery is an efficient and modern way of delivery in tissues and in tissue engineering processes [27, 28]. Drug delivery and tissue engineering have some similar requirements, as both drug delivery vehicles and tissue engineering scaffolds need to be biocompatible and biodegradable, properties which can be well met with the aid of the electrospinning process [26]. Electrospun nanofibers are the most widely used carriers of biomolecules and have many advantages, including sustained drug release, high efficiency of drug loading, flexibility in shape, high surface-to-volume ratio, and high porosity [27]. Because of their specific characteristics, these NFs are extensively utilized in drug delivery in treating different disorders [22].

## 2. Inorganic Materials

Inorganic materials including metals, surface-treated/ceramic-coated metals, and bioactive ceramics (particularly calcium phosphate ceramics) have been widely used in bone tissue engineering and actively bind to the bone. Since the bone composition is mainly of type I collagen and inorganic crystals of carbonate-substituted HA (a basic calcium component), those implanted surfaces containing such materials (synthetic HA) will reveal osteoinductive properties. Adding these materials to electrospun NFs will improve the adhesion and differentiation of cells. This was shown in a study where after adding collagen/n-HA to PLGA NFs increased osseointegration and bone regeneration [26]. In addition, inorganic nanoparticles (NPs) like halloysite nanotubes (HNTs), carbon nanotubes (CNTs), graphene, nanohydroxyapatite (n-HA), Laponite ® (LAP), and mesoporous silica (MMS) are widely used because of their high surface ratio and higher drug-loading capacity. These NPs are biocompatible and promote cell functionality that can make them useful in tissue engineering. As an example, a study showed that nanosilicate (nSi) has a high degree of effectiveness in promoting bone healing [29]. However, studies showed that combining these inorganic NPs with electrospun nanofibers (NFs), thereby creating a hybrid of organic/inorganic NFs, revealed improved drug loading and cellular response, which makes them more useful in both drug delivery and tissue engineering application. On the other hand, inorganic NP loading in nanofibers significantly increased NFs mechanical properties, cell adhesion, migration, proliferation, and differentiation. These hybrid NFs prolong drug release and inhibit burst release of drugs, with application as an antibiotic and in cancer drug delivery. As an example, some antibiotic drugs such as amoxicillin (AMX) and tetracycline hydrochloride (TCH) can be formulated as organic/inorganic NFs. In addition, anticancer drugs can be loaded in these hybrid forms. One such cancer drug which has been widely studied is doxorubicin (DOX), where the hybrid formulation sustainably releases the drug [30]. Recently, nanotechnology and nanoscience-based organic-inorganic composites are developed to expand the market in tissue engineering [26]. However, these kinds of scale-up formulation studies are limited; therefore, to find out more about their safety and stability, in vivo studies should be done in preparation for clinical trials [30].

Currently, several statin nanofibers have been synthesized for different purposes, especially bone regeneration and endothelial stenosis reduction. We have reviewed literature studies and identified a number of studies related to the clinical application of statin nanofibers. We review and summarize a number of such studies here.

## 3. Bone Application

### 3.1. In Vitro

Kalani et al. evaluated the osteogenesis differentiation of human adipose-derived stem cells (hADSCs). To this purpose, they prepared slow-release core-sheath poly(vinyl alcohol)/silk fibroin nanofibers (PVA-SF core-shell NFs) with rosuvastatin (RSV) by a coaxial electrospinning process. After culturing the hADSCs on RSV-loaded NFs, these NFs have significantly upregulated osteogenesis markers such as Col 1, RUNX2, alkaline phosphatase (ALP) (two early osteogenesis markers), and osteocalcin (OCN) (a late osteogenesis marker) compared to free-drug NFs. Also, ARS staining confirmed the osteogenesis by showing calcium formation. Therefore, the PVA-SF core-shell NFs, with sustained release of RSV, provide suitable applications in bone tissue engineering [31]. In another study by Kalani et al., RSV has been immobilized on silk fibroin (SF) NFs with the aid of an Argon Plasma method. The SF-RSV-P3, after 3 minutes of treatment with plasma, induced hADSCs proliferation and osteogenic differentiation more than all other formulations. In confirmation, proliferation and expression of Col1, RUNX2, ALP, and OCN were seen more in the case of the SF-RSV-P3 group. In addition, ARS staining showed the greatest calcium formation, attributed to higher RSV release from SF-RSV-P3 [31]. Furthermore, Rezk et al. in another study revealed that their novel formulation (functional composite nanofibers (FCNs)), which was loaded with beta-tricalcium phosphate (*β*-TCP) and simvastatin (SIM), showed better bone regeneration in comparison to the control group (pure NFs) with sustained drug release [32]. Another study by Rezk et al. produced SIM in a different formulation of a composite formulation of poly(*ε*-caprolactone) (PCL) and poly(glycerol sebacate) (PGS) loaded with hydroxyapatite nanoparticles (HANPs) and simvastatin (SIM) (PCL-PGS-HA-SIM). This study revealed that the presence of SIM increased MC3T3-E1 osteoblast cell proliferation rate more in comparison to that of PCL-PGS and PCL-PGS-HA, which was confirmed via kit-8 (CCK-8) assay. Also, PCL-PGS-HA-SIM showed improved cell adhesion and bone extracellular matrix (ECM) secretion after 6 days compared to PCL-PGS and PCL-PGS-HA [33] (Figure 1). Moreover, Rezk et al. produced another SIM formulation of PCL-NFs loaded with polyaniline-coated titanium oxide nanoparticles (TiO_2_/PANI) and SIM (PCL-PTS) using the electrospinning method. PCL-PTS showed the most MC3T3-E1 proliferation after 5 days, compared to the similar proliferation rates in all the different samples taken. PCL-PTS releases SIM gradually in a controlled manner within the first 5 days, beyond which SIM concentration and consequently cell proliferation increase simultaneously. All formulations in this study (PCL-PT, PCL-1PTS, PCL-3PTS, and PCL-5PTS) showed a significant adhesion rate and an increase in ECM rates, demonstrating successful mineralization, after 5 days [33]. In addition, in another study in [32], composite PCL/HA/simvastatin electrospun nanofibers (PCLHSs) were devised by coating them on biodegradable Mg alloy. In this study, CCK assay data showed that PCLHS had the highest cell proliferation rate amongst other samples, which again reveals the osteogenesis effect of simvastatin. Also, SEM findings showed that MC3T3 mouse osteoblast cell attachment was the highest in the PCLHS group, indicating that this formulation is a biocompatible candidate for bone regeneration [32].

### 3.2. In Vivo

Chitosan nanofiber membranes, with or without simvastatin, showed acceptable bone regenerations in rat calvarial defects. The results from the study showed no significant difference between the control and experimental groups in bone regeneration, and therefore, more studies still need to be performed [35]. Another study tested novel NF scaffolds on calvarial defects in rats. Simvastatin-loaded electrospun spiral-wound PCL scaffolds after 3–6 months significantly reconstructed the 8 mm calvarial defect with an increased mineralization rate compared to free PCL scaffolds. Although PCL scaffolds do promote bone mineralization, they are however generally limited to nonhealing in extent [36] (Figure 2). Employing the “Simvastatin-Releasing, Biodegradable, Nano to Microscale Fiber Scaffold (SRBFS)” promoted considerably higher bone formation than the free scaffolds (BFS) after 12 weeks of implantation in mice. This was further confirmed by the rate of calcium deposition and ALP activity, which were comparatively higher in the SRBFS group [37]. In the study by Hajializade et al., simvastatin and/or ezetimibe-loaded polyurethane (PU) nanofibers showed significant bone healing and increased bone density in a 5–7 mm femoral defect in rats. Amongst the three formulations, combination of simvastatin and ezetimibe nanofibers showed the highest bone density and healing effects [22].

## 4. Endothelial Stenosis and Thrombosis

### 4.1. In Vitro

A study by Chu et al. evaluated the proliferation and attachment efficacy of atorvastatin calcium (AtvCa) embedded in poly(L-lactide-co-caprolactone) (PLCL) nanofiber-covered stents within vascular endothelial cells (HUVECs). The study revealed that these NFs showed controlled release and could induce HUVEC proliferation in a dose-dependent manner. The effect was dependent on concentration, as with 5 ± 1 nM of AtvCa or PLCL-AtvCa10 nanofiber, HUVEC proliferation was increased, whereas with 12 nM AtvCa, it decreased [38] (Figure 3).

A heparin-rosuvastatin (Rosu)-loaded P(LLA-CL) nanofiber-covered stent tested in smooth muscle cells (SMCs) showed that by increasing the Rosu concentration, the SMC proliferation decreased [39]. Another study by Liu et al. used a new rosuvastatin calcium and heparin-loaded PLCL scaffold, comprising a core solution of 150 mg/mL heparin and 10 mg/mL rosuvastatin. The volume ratios of heparin-to-rosuvastatin calcium solution were 450 : 50 mL (Rosu 50), 425 : 75 mL (Rosu 75), and 400 : 100 mL (Rosu 100). Between these, Rosu 75 and Rosu 100 demonstrated significant anticoagulation and RBC attachment inhibition. In this study, a rabbit aneurysm model was created and DSA followed up after 4 months revealed that aneurysms disappeared slowly in all Rosu groups. Rosu 100 showed the best reendothelization and intima coverage results amongst its counterparts (covered stents). In addition, it was also discovered that rosuvastatin normally increased the VEGF-A levels [40]. In a recent study conducted by Feng et al., a novel stent covered with heparin and rosuvastatin calcium-loaded P(LLA-CL) nanofibers was tested for the treatment of aneurysm. CCK-8 assay was used for evaluating the proliferation and adhesion rates of HUVECs, which after 36 hours reported better proliferation and adhesion for Rosu 75 and Rosu 100 than Rosu 50 and free-drug NFs. Moreover, Rosu 100 promoted the best anticoagulation ability. As both heparin and rosuvastatin have anticoagulation ability, a synergistic effect results in these formulations [41]. Lee et al. produced novel bifurcation stents coated with bio-absorbable nanofibers loaded with rosuvastatin and paclitaxel. These stents show two different mechanisms: firstly, rosuvastatin decreased the platelet adhesion, while the paclitaxel acts by inhibiting SMC proliferation [42].

### 4.2. In Vivo

In a DSA follow-up study with a rabbit aneurysm model, aneurysms completely disappeared after one month of administration. All atorvastatin calcium (AtvCa) in the PLCL nanofiber-covered stents was fully embedded on the artery, with the exception of PLCL-AtvCa5. Among the various formulations, PLCL-AtvCa10 gave the best results, including reendothelization and intimal hyperplasia [38].

In the study by Liu et al., an aneurysm was induced in the right common carotid artery (CCA) of the rabbit. A heparin-rosuvastatin-loaded P(LLA-CL) nanofiber-covered stent was then placed on the aneurysms. The DSA follow-up showed that after 30 days, aneurysms decreased and gradually disappeared. No stenosis in the CCAs was found in either the short- or long-term follow-ups. This was also seen among different formulations. The best effectiveness in reducing in-stent stenosis and thrombosis was shown by Rosu 100 with 15% heparin and 20 *μ*M rosuvastatin solution (400 : 100 *μ*L) [39] (Figure 4).

## 5. Anti-Inflammatory Effect

### 5.1. In Vitro

A study by Schwinte ´et al. developed a nanofibrous polymeric membrane bearing nanocontainers of atorvastatin complexes to validate anti-inflammatory effects. For this purpose, free and statin PCLs seeded on control and LPS-stimulated THP-1 cell cultures were employed and their anti-inflammatory effect was monitored for 6–48 hours. The results from this experiment demonstrated that both TNF-*α* and IL-6 secretions decreased in AT-PCL NFs, with TNF-*α* showing an inhibition of about 60% at 48 h independent of dose and IL-6 showing >80%, which decreased in a dose-dependent manner [43].

## 6. Neuroprotective Effect

### 6.1. In Vivo

Peripheral nerve injury (PNI) treatment has remained a serious medical problem till date. A sciatic nerve crush injury rat model was used by Haidar et al. to validate the efficacy of composite nanofibers incorporating alpha lipoic acid (ALA) and atorvastatin (ATR) (Figure 5). They evaluated different factors to assess functional and sensory recovery in rats. The authors considered that Sciatic Functional Index (SFI), BBB score, Extensor Postural Thrust Test (EPT), Withdrawal Reflex Latency (WRL), ultrastructural examination, and measures of TNF-*α*, IL-1*β*, and IL-6 levels showed better results for the ALA/ATR group than other formulations and the control group. Also, it should be mentioned that all ATR groups suppressed the inflammation factors well [44].

## 7. Conclusion

Herein, studies related to various in vitro (Table 1) and in vivo (Table 2) applications of statin nanofibers have been reviewed, and the results of such studies are summarized. The resulting search indicates that the applications of statin nanofibers pertain to thrombosis, bone regenerative, and endothelial stenosis, along with anti-inflammatory and neuroprotective effects which were also identified in two different studies.

For bone regeneration, simvastatin and rosuvastatin in in vitro studies applied to two different cell lines hADSCs and MC3T3-E1 showed induction of cell proliferation, adhesion, and osteogenesis differentiation. Furthermore, in vivo studies in which simvastatin nanofibers were applied to calvarial or femoral defects revealed bone healing ability, with one exception. This particular study showed no difference between the statin nanofiber and free polymer nanofiber, and further investigation needs to be done.

In vitro studies in the field of endothelial stenosis and thrombosis demonstrated that atorvastatin and rosuvastatin NFs-covered stents caused HUVEC proliferation and adhesion in a dose-dependent manner. In one study, a low dose (5 ± 1 nM) of AtvCa increased proliferation, whereas at a higher dose (12 nM), HUVEC proliferation decreased. Addition of an anticoagulant agent like heparin to the formulation showed a synergistic effect. Moreover, addition of paclitaxel showed inhibition in SMC proliferation. Reduction of SMC proliferation, anticoagulation, RBC attachment inhibition, reendothelization, and intima coverage increased VEGF-A levels, with simultaneous decrease in platelet adhesion. This was confirmed from other in vitro findings, which overall confirm the antithrombosis and reendothelization actions. In all in vivo studies in rabbits, where CCA aneurysm was induced, disappearance of the clot was observed at particular time durations.

One study on atorvastatin NFs revealed that anti-inflammatory effect of these agents is related to the decrease in both TNF-*α* and IL-6 secretions. While the reduction of IL-6 occurred in a dose-dependent manner, TNF-*α* reduction was not dose related. This anti-inflammatory effect is also detected in some endothelial stenosis and bone regeneration studies.

Finally, experiments involving peripheral nerve injuries like sciatic nerve crush have also been treated by a NF formulation containing atorvastatin and ALA.

Following these studies, it can be concluded that statin NFs, specifically atorvastatin, simvastatin, and rosuvastatin, are effective in healing bone fracture, aneurysm, and sciatic nerve crush as a result of their sustained drug release profile, although clinical trials still need to be performed to confirm these data. Therefore, these collective results reveal that statins are pleiotropic agents that are effective in various different fields apart from hypercholesterolemia. In addition, more studies are still needed to discover new applications of these promising agents.

## Figures and Tables

**Figure 1:** Preparation of nanofibers with the electrospinning method and the osteogenesis in vitro process; reproduced from [33], with permission from [34].

**Figure 2:** Micro-CT 3D images representing whole sample: ‘‘simvastatin-containing PCL scaffolds”; PCL scaffold without simvastatin; ‘‘simvastatin-embedded PCL scaffolds”; and critical size defect without any scaffold (control group). (a) 3 months and (b) 6 months; reproduced with permission from [36].

**Figure 3:** (a) HUVEC migration in different nanofiber film environments after 6, 12, and 24 hours and (b) micrographs stained by crystal violet. (c) The NO release of HUVECs on different nanofiber films and (d) micrographs of fluorophore probe DAF-FMDA. ^*∗*^Significant difference of *p* < 0.05; reproduced with permission from [38].

**Figure 4:** (a) Schematic illustration showing the creation of the rabbit aneurysm model and a photograph showing aneurysm (arrow) formation during operation. (b) Schematic illustration showing aneurysm formation and an angiograph showing aneurysm (arrow). (c) Schematic illustration and an angiograph showing aneurysm closure after stent implantation. (d) Angiograph illustration types A, B, and C in the long-term follow-up. Bar graph showing the number of different types in the Rosu 100 group vs the PBS group; reproduced with permission from [40].

**Figure 5:** In vivo animal model for peripheral nerve injury on the sciatic nerve (a). A healthy sciatic nerve after surgical splitting of the muscles (b). Application of the Yasargil aneurism clip for trauma on the sciatic nerve (c). The sciatic nerve injury site after removal of the Yasargil aneurism clip (d). Implantation of composite nanofibers around the injured sciatic nerve just after the trauma (e). Scanning electron microscopy images of (e). Composite nanofibers containing ALA- and ATR-loaded chitosan nanoparticles (f). ATR-loaded chitosan nanoparticles existing in the composite nanofiber structure; reproduced with permission from [44].

**Table 1:** Summary of in vitro applications of statins in various studies.

Application	Reference	Cell line	Product	Authors' stated main result
Bone regeneration	[32]	MC3T3 mouse osteoblast cell line	Composite PCLHS coated on biodegradable Mg alloy	PCLHS-NFs increase both bone regeneration and control its degradation
	[45]	-	FCN loaded with *β*-TCP-SIM-NFMS	FCN-*β*-TCP-SIM-NFMs revealed better cell proliferation and attachment than the control fiber
	[33]	MC3T3-E1 osteoblast cells	PGS-HA-SIM composite NFs	PCL-PGS-HA-NFs are suitable for both increasing bone tissue regeneration and controlled drug release
	[46]	MC3T3-E1	PCL-PTS-NFs	PCL-PTS-NFs both cause controlled drug release and increase cell regeneration and adhesion compared to the control group (PCL)
	[31]	Human adipose-derived stem cells (hADSCs)	PVA-SF core-shell NFs with RSV	PVA-SF core-shell NFs with RSV increased cell proliferation and osteogenic differentiation
	[47]	Human adipose-derived stem cells (hADSCs)	SF-RSV-P3-NFs	SF-RSV-P3 with RSV sustained release enhanced osteogenesis

Endothelization and antithrombotic effects	[48]	Vascular endothelial cells (HUVECs)	AtvCa in the inner of PLCL-NFs-covered stents	AtvCa-PLCL-controlled release NFs-covered stents cause HUVEC proliferation in a dose-dependent manner
	[39]	Smooth muscle cells (SMCs)	A heparin-Rosu-loaded P(LLA-CL) NF-covered stent	The heparin-Rosu-loaded P(LLA-CL) NF-covered stent declined SMC proliferation with enhancement of Rosu concentration
	[40]	Rabbit aneurysm model	Rosu-calcium-heparin-loaded PLCL scaffold	Rosu 100 exhibited the best reendothelization and intima coverage results among all other covered stents
	[41]	HUVECs	Heparin-Rosu-calcium-loaded P(LLA-CL) NFs-covered stents	Heparin-Rosu-calcium-loaded P(LLA-CL) NFs shows a significant anticoagulation ability
	[42]	SMCs	Rosu-paclitaxel-NFs bifurcation stents	The Rosu-paclitaxel-NF-covered stent declined SMC proliferation and platelets adhesion

Anti-inflammation	[43]	THP-1 cell culture	Atorvastatin-PCL NFs	Atorvastatin-PCL NFs of 60% inhibited TNF-*α* and 80% inhibited IL-6

**Table 2:** Summary of in vivo application of statins in various studies.

Application	Reference	Animal model	Lesion type	Product	Dose	Treatment duration	Authors' stated main results
Bone regeneration	[35]	Sprague-Dawley rats	Rat calvarial defects	Chitosan with or without SIM-loaded NFMs	0.25 mg of simvastatin	8 weeks	There was no significant difference between the control and experimental groups
	[36]	Wistar albino rats	Rat calvarial defects	SIM-loaded electrospun spiral-wound PCL scaffolds	20 *μ*g	6 months	The SIM NFs after 3–6 months significantly reconstructed the 8 mm calvarial defect with increase in the mineralization rate compared to free PCL scaffolds
	[37]	Mice (C57/bl/6j, 4 weeks old, male)	Bilateral dorsal skin	SRBFS	0.025 wt%	12 weeks	SRBFS promoted substantially higher bone formation than the free scaffolds (BFS) after 12 weeks of implantation on mice.
	[22]	Wistar rats	5–7 mm femoral defect	SIM and/or ezetimibe-loaded-PU-NFs	0.471 mg/oval fracture shape	4 weeks	SIM and/or ezetimibe-loaded PU-NFs showed significant bone curing and increased bone density

Endothelization and antithrombotic effects	[38]	Rabbit aneurysm model	Intracranial aneurysm in a rabbit carotid artery aneurysm	AtvCa in the inner of PLCL-NFs-covered stents	5, 10, 15, and 20 mg	One month	Aneurysms completely disappeared; PLCL-AtvCa10 showed the best results, including reendothelization and intimal hyperplasia
	[39]	Rabbit aneurysm model	Rabbit right CCA aneurysm	A heparin-Rosu-P(LLA-CL) NF-covered stent	10 mg/mL rosuvastatin	4 months	Among different formulations, Rosu 100 showed the best effectiveness in reducing in-stent stenosis and thrombosis

Neuroprotection	[44]	Sprague-Dawley male rats	Sciatic nerve crush injury	ALA-ATR composite NFs	-	One month	ALA/ATR showed better results than other formulations

## Data Availability

No data were used to support this review article.
